# Monitoring and Analysis Solid Formulation Dissolution Phenomenon with Image Recognition Technologies

**DOI:** 10.1155/2022/3997870

**Published:** 2022-09-14

**Authors:** Haoyu Wang, Chiew Foong Kwong, Qianyu Liu, Junyao Liu, Zhixin Liu, Boon Giin Lee, Liang Huang

**Affiliations:** ^1^Department of Electrical and Electronic Engineering, University of Nottingham Ningbo China, Ningbo, China; ^2^Next Generation Internet of Everything (NGIoE) Laboratory, University of Nottingham Ningbo China, Ningbo, China; ^3^School of Information Science and Engineering, NingboTech University, Ningbo, China; ^4^Central Research Institute, Shanghai Pharmaceutical Holding Co., Ltd., Shanghai, China; ^5^Department of Outpatient, Liaoning Blood Embolus Medical Centre, Shenyang, China; ^6^Department of Computer Science, University of Nottingham Ningbo China, Ningbo, China

## Abstract

The dissolution test has become the most important quality index in the research and development of solid formulation, especially the evaluation of drug bioequivalence. However, it had low operability, was tedious, and was always overlooked. The previously related studies required a fixed tablet and analysed the recorded video by disso GUARO PRO and Microsoft Paint™. Therefore, we have developed a novel image recognition system to automatically track the moving tablet and analyse the volume change at the same time. Image recognition technology is often used to monitor the dissolution process. The camera system with visible light and infrared camera functions was placed on the dissolution tester. The system collects the plate image for binary processing and then records and calculates its pixel area, which can automatically record the volume change of the tablet in the dissolution test, no matter disintegration or corrosion.

## 1. Introduction

Image recognition technology is an important tool to monitor different experimental phenomena in the absence of experimental personnel. Recording and analysis of dissolution test videos are for studying tablet behavior during the dissolution test. In Felicijan's study [1], an iron wire was used to fix the tablet at the bottom of the dissolution cup. Then, a 10-second video of the dissolution process was recorded at each sampling point. After that, the video is fed into software named *disso GUARO PRO* to reduce the noise of particles in the dissolution liquid before Microsoft Paint™ calculates the relative volume of the tablet. A red-light source was used to record photo instability tablets. The fixed tablet can provide a stable image to capture but may influence the dissolution result. Besides, real-time monitoring cannot be realized by recording the video and then entering it into other software, which also makes monitoring more complicated. The red-light source can basically solve the recording of photo instability tablet behavior, but infrared ray with lower light particle energy is a better choice. Li et al. [2] also use a camera to record the dissolution test. Morita et al. [3] chose three tablets to calculate the trim size of tablets, which were fixed at the bottom of the dissolution cup by an iron wire. A camera on the top of the dissolution cup recorded the changes on the surface of these three tablets, and the space between these three tablets was used to calculate the area changes on the tablet surface. Nevertheless, based on the guidance of drug administration in all countries, both tablet fixing and multitablet dissolution tests were limited. Chinese patents 201721009959 [4] were focused on carrying out the overall design of the monitoring dissolution equipment. However, its function is relatively simple, only with real-time monitoring and video recording functions. In addition, these two designs are also unable to monitor the dissolution appearance of photolabile drugs under night vision. Kazarian and van der Weerd [5] used simultaneous macrophotography and Fourier transform infrared spectroscopy attenuated total reflection (FTIR-ATR) imaging to explain the physical changes of hydroxypropyl methylcellulose (HPMC) andBuflomedil pyridine phosphate tablet during the lysis of the specially designed cells. By utilizing macrophotography alone, the changes in tablet appearance can be observed, but the substance concentrations cannot be quantified. However, by employing FTIR-ATR imaging simultaneously, both water immersion and drug concentration at different locations of the tablet were quantified, thus showing the relationship between the visually observed fronts (i.e., gel formation front and erosion front) and different yields of water. Morita et al. [6] also analyzed the disintegration time of rapidly disintegrating tablets by means of a camera. Treacher et al. [7] adopted photographic images of the dissolution process in specially designed flow cells to observe the tablets containing varying amounts of felodipine, a drug that is less soluble in water. Specifically, the tablets with small drug content dissolved completely while, with regard to the tablets with large drug content, they had the same appearance before dissolution but decreased in tablet size after initial swelling. Cao et al. [8] investigated the changes in the photographic image over time during the release study of HPMC-coated tablets by using a camera on the side of the dissolution vessel in a USP paddle apparatus. The initial swelling of the photographic images and the subsequent disintegration of the coating tablet were related to good drug release. Tieu et al. [9] made use of a camera to provide the side and bottom views of the dissolution vessel so as to assess different potentials for monitoring the dissolution process via video. Moreover, it was concluded that the camera could easily evaluate the presence or absence of a tablet and its location in the dissolution vessel. In addition, they not only suggested utilizing the cameras during the preparation of the formula but also studied the camera recordings of the dissolution systems for different vessels and vessel heating types, as well as different camera angles, so as to evaluate the use of video surveillance in several devices.

The drug release process is controlled by two mechanisms of dissolving drugs, namely disintegration and erosion, which often occur simultaneously [10–12]. Drug solubility affects gel properties, and drug release and poorly soluble drugs reduce the entanglement of the polymer chains, thus reducing the gel strength [13, 14]. Therefore, erosion becomes the main release mechanism. Regarding the highly soluble drugs, the release from the matrix is believed to be primarily diffusion-controlled. Furthermore, the highly soluble drugs may act as pore former in the gel, thus enhancing the perviousness of water. Moreover, they can be regarded as additional permeability contributors, thus increasing the growth of the gel layer [15].

The purpose of this study is to offer a dissolution phenomenon behavior system by using image recognition to record videos and use the pixel area to calculate the tablet volume change. Besides, the model can also automatically trace the tablet. Based on the volume change of disintegration and corrosion phenomenon, the system uses the decision tree method to give the results of phenomena. In order to solve the problem of recording the phenomenon of light unstable drugs, the camera in the system has the function of recording under infrared light. Also, some infrared lights are installed on the camera.

## 2. Materials and Methods

### 2.1. Materials

Albendazole tablets 200 mg/tablet (Sino-American Tianjin Skincare Pharmaceutical Co., LTD.), Famotidine tablets 20 mg/tablet (Guangdong Bidi Pharmaceutical Co., LTD.), and lemon mints were used in this study.

### 2.2. Dissolution Studies

A Huanghai RCZ-1B (Shanghai Huanghai) dissolution tester with a paddle method was used in this project.

The dissolution medium was pure water. A 900 ml dissolution medium was placed in a dissolution cup at 36.5 to 37.5°C. The speeding rate of the blade was set as 50 rap per minute. To monitor the drug dissolution phenomenon, the tablet volume change was recorded every 10 seconds.

### 2.3. Camera System

An IR-CUT camera with the function of both an infrared camera and a visible light camera achieved by an automatic switch was used to record the image day and night. 6 IR lights were installed on the camera to obtain a dark environment light source. Furthermore, a light-dependent resistor (LDR) was used to switch the IR and visible light modes. The photo of the IR-CUT camera and the structure of the IR-CUT camera system are shown in Figure 1.  Figure 2 shows an IR-CUT camera system structure chart.

As shown in Figure 1, 6 infrared light sources are posited on both the left and the right of the camera. A blue element besides the camera is the LDR.

As shown in Figure 2, the system is with an image analysis system (including hardware and software), infrared light source, camera, circuit board, and LDR.

Figure 3 is the whole instrument system structure chart with both software and hardware for the dissolution test. The instrument system contains an image analysis program, a computer, a dissolution tester, visible/infrared light sources, and an IR-CUT camera/normal camera. The image would be transferred into the image analysis program from the camera, and the scatter diagram would be output as a result after analysis.

### 2.4. Program Modeling

The following four steps are used to achieve image recognition [16 to 25] in the image analysis program.

#### 2.4.1. Get the Original Image

The first step is starting the program to call the camera and then get a frame of the image.

#### 2.4.2. Image Reprocessing

To improve the speed of image processing, the original image was resized. After that, box blur was used to remove the noise to achieve image contour connection.

#### 2.4.3. Image Segmentation

Image binarization is based on the threshold method with the tablet as white and the background as black. Then, the white hole was removed using morphological transformation, and the white area contour was found to calculate the relative area. The size of the white area was employed to judge whether it was a tablet. The “central point” of this contour was worked out using the average method, which set the average *x*-axis of the top point and bottom point as the “central point” *x*-axis and the average *y*-axis of the left point and right point as the “central point” *y*-axis, with the contour as the target tablet. Finally, the tablet's position was confirmed after the region grows based on the “central point.”

#### 2.4.4. Data Visualization

According to the pixel of the region growth image, the relative area of the tablet was calculated. A scatter diagram with a trend line was plotted in real time.

Figure 4 shows the whole process of this program.

## 3. Result and Discussion

To determine the influence of different tablets, a classification method was proposed in this section. Based on their appearance, tablets can be divided into big tablets, small tablets, and tablets with different colours. Disintegration and corrosion are two standards of classification of the dissolution phenomenon. Moreover, an infrared light camera was used to solve the stable problem of light-sensitive tablets. In this section, experimental was designed to test the adaptability in this condition.

### 3.1. Disintegration Tablet Image Recognition Test

The program suitability tests for disintegrating tablets are divided into big-volume tablets and small-volume tablets.

Big-volume tablets: since the inactive ingredients in big volume tablets are insoluble in water, they will suspend in the liquid under the action of the paddle. Due to the overmuch insoluble ingredients of big volume tablets, the dissolution medium will become cloudy until it is invisible to the naked eye in the disintegration process. Consequently, the resolution ability of the program in the case of noise interference needs to be tested with big-volume tablets as the test standard. If the high-dose tablets are successful, the system could meet most of the experimental requirements.

Small-volume tablets: small-volume tablets are the limit test for the resolution of the system. Since the recognition of tablets in the system is based on area, the system may ignore small-volume tablets. This experiment uses small-volume tablets for limit testing. If there is a good result of the test, it means that the system's adaptability to tablet volume can meet the needs of routine experiments.

#### 3.1.1. Big Size Disintegration Tablets

Sample: albendazole tablets 200 mg/tablet (Sino-American Tianjin Skincare Pharmaceutical Co., LTD.)

Appearance: a white-coated round medicine, white or similar white after removing the coating.

According to the analysis of its prescription, this formulation conforms to the characteristics of the samples required in this experiment. The experimental results are shown in Figures 5–7 as follows. Each group of figures consists of three figures. The first image is a scatter diagram of volume changes over time and a real-time trend line. The unit of the horizontal axis is seconds, and the vertical axis is in pixels. The second figure shows a screenshot of the actual tablet, and the third figure is the image after binarization.

As shown in Figure 5, after the tablets were put in, the system started to identify the tablets, draw a scatter diagram of the area of each period according to the pixel area and dynamically add a trend line to guide the observation according to the trend scatter.

As shown in Figure 6, the tablets start to absorb water and get imbibition, appearing like a cake shape. At the same time, the process of disintegration begins. According to the curve and scatter diagram, the trend of the volume can be judged.

As shown in Figure 7, consistent with the trend line, it can be found that its volume becomes stable after 200 seconds, indicating the disintegration phenomenon completed at the same time. The remaining identification images are all conical precipitates formed by water-insoluble inactive ingredients.

According to Figures 5–7, the liquid in the dissolution cup at the end of the disintegration process is very turbid, which is almost indistinguishable by the naked eye. However, the system can still effectively identify the aggregated objects, indicating that it could be employed in practical applications. In conclusion, it can replace the experimenter to observe the dissolution behaviour of big-volume tablets.

#### 3.1.2. Small Size Disintegration Tablets

Sample: famotidine tablets 20 mg/tablet (Guangdong Bidi Pharmaceutical Co., LTD.)

Appearance: white and round tablet.

The experimental results are shown in Figures 8–10. Each group of figures consists of three figures. The first image is a scatter diagram of volume changes over time and a real-time trend line. The horizontal axis is in seconds, and the vertical axis is in pixels. The second figure shows a screenshot of the actual tablet, and the third figure is a binarized image.

As shown in Figure 8, after the small tablet is put into the dissolution cup, the image recognition program successfully recognizes them and starts to draw a scatter diagram of area changes.

Figure 9 shows that the small tablet starts to absorb water and get imbibition. After that, particles spread in every part of the dissolution medium, but the image recognition program still clearly recognizes the tablet and paints an exemplary scatter diagram.

The completion of small-volume tablet disintegration is shown in Figure 10, and most of the insoluble particles are suspended in the cup. Since the particles are smaller than the set limit value, they are no longer recognized. According to the final curve, the area change of the whole dissolution process can be observed easily.

Since the particles are below the set limit value, they were no longer recognized. According to the final curve, the area change of the whole dissolution process can be observed easily.

This experiment examined the system's ability to recognize small-volume tablets, which turned out to meet the needs of typical experiments.

#### 3.1.3. Erosion Tablets

The erosion phenomenon usually occurs in the dissolution experiments of standard formulations and sustained-release formulations with dissolution skeletons. Among them, two widely recognized soluble formulations are candy and lozenges. The sample used here is a lemon mint tablet with yellow colour and double-layer structure.

The experimental results are shown in Figure 11. Each group of figures consists of three figures. The first image is a scatter diagram of volume changes over time and a real-time trend line. The horizontal axis is in seconds, and the vertical axis is in pixels. The second figure shows a screenshot of the actual tablet, and the third figure is the image after binarization.

Figure 11 shows that the tablets are placed at the bottom of the dissolution cup, the image recognition program starts to identify them effectively, records the scatter diagram of volume changes, and adds the real-time trend line.

As shown in Figure 12, the tablet gradually dissolved and became smaller in size. The image recognition program is also operating normally, the scatter diagram is plotted well, and the real-time trend line goes well.

As shown in Figure 13, due to the fragmentation phenomenon of the tablet during the dissolution process, resulting from the data and the scatter diagram anomaly, but as the fragments continue to become smaller, the data return to the trustworthy interval.

As shown in Figure 14, the tablet has been completely dissolved. According to the scatter diagram, the volume (recognition area) changes during the eroding period can be accurately analyzed.

In this dissolution experiment, unexpected situations (such as tablet debris) may cause short-term analysis errors. However, as the large pieces of debris gradually became smaller, the system returned to normal and accurately depicted the scattered points of the identified area image and reasonably added real-time trend lines.

#### 3.1.4. Different Colour Tablets

The coating of tablets has a variety of colours.  Figure 15 shows the coating colour card provided by Shanghai Colorcon Coating Technology Co. Ltd. There are 200 colours from dark to light, which is undoubtedly a challenge to the sensitivity of image recognition in the dissolution experiment.

In order to increase and test the adaptability of the system, we selected white, yellow, bright red, bright blue, deep blue, dark red, green, and purple small round plastic plates to test the recognition ability of the system. Eight groups of figures are shown in Figures 16–23.

The first figure shows an actual photo of each set of plastic sheets. Moreover, the second figure is the photo of the plastic plates at the bottom of the dissolution cup. The image after binarization is shown in the third figure. The fourth figure shows the photo after noise cancellation.

In this test, eight colours covered the spectrum from long optical to short optical wavelength and received a good result that the image recognition program can successfully recognize these colour plates. It means that the program has suitable suitability in tablets with standard colours.

#### 3.1.5. Infrared Condition

For some photosensitive drugs, the dissolution experiment needs to do shading treatment. Visible light cameras cannot be used because the water bath completely blocks light. Consequently, the infrared camera is recruited to make up for the deficiency. In addition, the image recognition of the infrared camera was optimized in this system. The advantage of infrared cameras is not just that they can be used without visible light. The images are usually black and white, so in this experiment, the colour of the tablet is not a factor. This system used the IR-CUT camera module, with the main structure as an LDR to control the switch between the infrared camera and the visible camera. Six infrared light sources automatically turn on when the camera is switched into the infrared camera mode, infrared mode, and visible light mode. Figures 24–26 are the system practicability test of the infrared camera under an infrared light source. The sample used in this experiment is the same as those used in the small volume tablet experiment.

The first image is a scatter diagram of volume changes over time and a real-time trend line. The unit of the horizontal axis is seconds, and the vertical axis is in pixels. The second figure shows a screenshot of the actual tablet, and the third figure is the image after binarization.

As shown in Figure 24, when the tablet is located at the bottom of the dissolution cup, the infrared camera successfully captures the tablet, and the image recognition program successfully recognizes it.

As shown in Figure 25, the tablet begins to absorb water and expand. At the same time, the reflection of the stirring paddle in the second figure did not interfere with the image recognition shown in the third figure. The program runs good and plots the ideal scatter diagram, and real-time trend lines are added.

As shown in Figure 26, the disintegration of the tablet is completed, and the water-insoluble inactive ingredients precipitate and accumulate. As shown in the scatter diagram in the first figure, after about 300 seconds, the area tends to be constant. As a result, the total disintegration time can be judged at about 300 seconds based on the scatter diagram and the trend line.

As a result, a summarized table is shown in Table 1 as follows.

## 4. Conclusion

This paper shows that the real-time dissolution phenomenon monitoring (RTDPM) system provides a solution to capture the moving tablets and provides a camera system to reduce the risk of light unstable tablets. This has been proven in the tests where it can satisfy the disintegration phenomenon of both small and regular-size tablets. Besides, the volume change curve of the corrosion plate can also be recorded. For some tablets that are less stable in visible light, the IR method can give a perfect solution (all substances above absolute zero emit infrared light. The infrared light source of the IR camera can slightly enhance the illumination intensity but not luminous energy). To sum up, this system can solve most dissolution test image recognition problems. However, the colour of the tablets and the light jam of the environment in this system still affect the test result, which should be noted in future research.

## Figures and Tables

**Figure 1:** The photo of the IR-CUT camera module.

**Figure 2:** An IR-CUT camera system structure chart.

**Figure 3:** The whole instrument system structure chart.

**Figure 4:** The image analysis program.

**Figure 5:** The experimental results of big size disintegration tablets (1).

**Figure 6:** The experimental results of big size disintegration tablets (2).

**Figure 7:** The experimental results of big size disintegration tablets (3).

**Figure 8:** The experimental results of small size disintegration tablets (1).

**Figure 9:** The experimental results of small size disintegration tablets (2).

**Figure 10:** The experimental results of small size disintegration tablets (3).

**Figure 11:** The experimental results of erosion tablets (1).

**Figure 12:** The experimental results of erosion tablets (2).

**Figure 13:** The experimental results of erosion tablets (3).

**Figure 14:** The experimental results of erosion tablets (4).

**Figure 15:** General color wheel from Shanghai Colorcon Coating Technology Co. Ltd.

**Figure 16:** White small round plastic plate.

**Figure 17:** Yellow small round plastic plate.

**Figure 18:** Bright red small round plastic plate.

**Figure 19:** Bright blue small round plastic plate.

**Figure 20:** Deep blue small round plastic plate.

**Figure 21:** Dark red small round plastic plate.

**Figure 22:** Green small round plastic plate.

**Figure 23:** Purple small round plastic plate.

**Figure 24:** System practicability test (1).

**Figure 25:** System practicability test (2).

**Figure 26:** System practicability test (3).

**Table 1:** A summarized table of experimental results and discussion.

Experiment	Results	Comment
Big volume tablet disintegration	According to the change in the measured area, the dissolution behavior was clearly recorded by the scatter diagram	N/A

Small volume tablet disintegration	The program successfully recognizes the small volume tablets from start to finish	N/A

Erosion	The output of the scatter diagram gives a trend of decreasing tablet volume	A short noise resulting from small tablet debris can influence scatter diagram plotting but not the trend line

Different colours	White, yellow, bright red, bright blue, deep blue, dark red, green, and purple small round plastic were used to test the applicability of white, and a good result was received	N/A

Infrared condition	Because of the stable light environment, the infrared condition experiment showed a good result	N/A

## Data Availability

The dataset can be accessed upon request.
